# Application of Multilayer Perceptron Genetic Algorithm Neural Network in Chinese-English Parallel Corpus Noise Processing

This article has been retracted.

**DOI:** 10.1155/2021/7144635

**Published:** 2021-12-20

**Authors:** Bing Li, Anxie Tuo, Hanyue Kong, Sujiao Liu, Jia Chen

**Affiliations:** ^1^College of Foreign Languages, Guizhou University, Guiyang 550025, China; ^2^College of Medical Humanities, Guizhou Medical University, Guiyang 550025, China; ^3^Guiyang No. 1 High School, Guiyang 550001, China; ^4^Department of Foreign Languages, Guizhou University of Traditional Chinese Medicine, Guiyang 550025, China

## Abstract

This paper uses neural network as a predictive model and genetic algorithm as an online optimization algorithm to simulate the noise processing of Chinese-English parallel corpus. At the same time, according to the powerful random global search mechanism of genetic algorithm, this paper studied the principle and process of noise processing in Chinese-English parallel corpus. Aiming at the task of identifying isolated words for unspecified persons, taking into account the inadequacies of the algorithms in standard genetic algorithms and neural networks, this paper proposes a fast algorithm for training the network using genetic algorithms. Through simulation calculations, different characteristic parameters, the number of training samples, background noise, and whether a specific person affects the recognition result were analyzed and discussed and compared with the traditional dynamic time comparison method. This paper introduces the idea of reinforcement learning, uses different reward mechanisms to solve the inconsistency of loss function and evaluation index measurement methods, and uses different decoding methods to alleviate the problem of exposure bias. It uses various simple genetic operations and the survival of the fittest selection mechanism to guide the learning process and determine the direction of the search, and it can search multiple regions in the solution space at the same time. In addition, it also has the advantage of not being restricted by the restrictive conditions of the search space (such as differentiable, continuous, and unimodal). At the same time, a method of using English subword vectors to initialize the parameters of the translation model is given. The research results show that the neural network recognition method based on genetic algorithm which is given in this paper shows its ability of quickly learning network weights and it is superior to the standard in all aspects. The performance of the algorithm in genetic algorithm and neural network, with high recognition rate and unique application advantages, can achieve a win-win of time and efficiency.

## 1. Introduction

Existing Chinese-English parallel corpus noise processing systems with high accuracy rate still have the disadvantages of time consumption, high cost, and inconvenient use [1]. The actual voice recognition system requires real-time Chinese-English parallel corpus noise processing on a general-purpose computer with limited resources [2]. Therefore, the development of fast recognition algorithms has been important in the study on noise processing of Chinese-English parallel corpora. Chinese-English parallel corpus noise processing technology is a subject that uses computers to analyze speech signals to realize automatic understanding of human speech [3]. Speech recognition technology has become a very active research field in information science. As a cross-discipline, it is gradually becoming a key technology of human-computer interaction in information technology [4]. Speech signal processing is a discipline that studies the use of digital signal processing techniques to deal with noise in Chinese-English parallel corpora. The purpose of processing is to obtain certain parameters for efficient transmission or storage or for certain applications, such as speech synthesis, Chinese-English parallel corpus noise processing, and speech enhancement. [5]. It is not only an effective and convenient way of information exchange, but also an important tool for humans to use machines. Whether it is the language communication between humans and machines, the noise processing of Chinese-English parallel corpus, especially the digital processing of voice signals, has a particularly important role [6]. Once voice recognition and voice synthesis technology are combined, people can leave the keyboard, receive voice commands, and perform operations [7].

Mohammad [8] proposed a neural network machine translation architecture, which is completely in terms of the neural network structure and is divided into two parts. The encoder converts the source language text into a set of context vectors and then decodes them. The processor then decodes the set of vectors into target language text. This structure completely gets rid of the previous statistical machine translation architecture. The model no longer includes explicit word alignment and translation rule extraction steps, which simplifies the complicated feature design work brought about by the complexity and change of natural language itself. With the attention mechanism proposed by Mojrian [9], the ability of neural network machine translation of processing long sentences has been further improved. The attention mechanism separately calculates the alignment information of the corresponding parts between the source sequence and the target sequence through weight distribution, so that the model “targets” the specified part in the training and prediction stages. Later, Lazli [10] and others further studied the attention mechanism, replacing the entire sentence with a fixed-length window, reducing the amount of calculation of this mechanism. The proposal of the attention force mechanism makes the results of neural network machine translation comparable to traditional statistical machine translation. As a result, neural network-based machine translation methods have become the mainstream method in the research field. At this stage, in order to overcome the gradient disappearance and gradient explosion problems that may be caused by the classic recurrent neural network model, the nodes of the network usually use complex structures such as LSTM (Long-Short Term Memory) and its variant GRU (Gated Recurrent Unit), so that model training is slow. Subsequently, in order to strengthen the accuracy of model training, Sheta [11] introduced a translation model based on convolutional neural networks, which uses convolutional neural networks to window and hierarchically extract sentence features, while retaining the accuracy of recurrent neural networks. Next, model training is accelerated through parallel computing. Poddar [12] realized the English-Chinese machine translation mode which is based on the sample neural network of the attention mechanism, using different Word2Vec models to generate English word vectors, and optimized the English-Chinese neural network machine translation model. Some scholars have implemented the machine translation model based on convolutional neural network and transformer-based English-Chinese machine translation model adding pretrained word vectors to the English-Chinese translation model and improving the quality of the model by providing prior information [13–15].

This article analyzes the specific content of neural networks and genetic algorithms on the basis of their respective shortcomings and analyzes the necessity and feasibility of combining neural networks and genetic algorithms. In the research of this article, by using the generation gap operator and the intersection operator based on the convex set theory, an improved genetic algorithm for the learning of neural network weights is formed, and the algorithm is used in the verification of the progressive voice. At the same time, the artificial neural network method can be helpful to design and implement the genetic algorithm. The impulse response or step response curve of the object is easier to obtain in the process. Take their series of values at the sampling moment as the information describing the dynamic characteristics of the object to form a predictive model. Because the nonparametric model is easier to obtain and the calculation is simple, the robustness is better. The structure and characteristics of the multilayer feedforward neural network are analyzed and summarized, as well as the computing power and function approximation of the multilayer feedforward neural network. Several methods for selecting the number of internal nodes and finally two heuristic algorithms and the implementation process are given: a detailed design of a genetic algorithm model is given, and related tests and performance analysis are done.

## 2. Chinese-English Parallel Corpus Noise Processing Model Based on Multilayer Perceptron Genetic Algorithm Neural Network

### 2.1. Multilayer Perceptron Hierarchical Distribution

Digital Chinese-English parallel corpus noise processing includes three aspects, namely, the digital representation method of Chinese-English parallel corpus noise, various methods and techniques of Chinese-English parallel corpus noise digital processing theory, and their practical applications in various fields [16].  Figure 1 shows the hierarchical spatial distribution of multilayer perceptrons.

For the corpus, the output value and expected output given by the neural network predictor for a period of time in the future are rolled to optimize the defined performance index function. After the training is over, the controller directly controls the controlled object. The basis of the noise parameter representation method is to regard the speech signal as the output generated by a certain model under a certain excitation and the excitation source and model. The parameter is used as a representation of the noise of the Chinese-English parallel corpus [17–19].

(1) $$\begin{array}{c} P\left(A,B\right)=P\left(A|B\right)\times P\left(B\right)=P\left(B|A\right)\times P\left(A\right),\\ E\left[{\left|Y\left(k\right)\right|}^{2}\right]=E\left[{\left|S\left(k\right)\right|}^{2}\right]+E\left[{\left|D\left(k\right)\right|}^{2}\right]. \end{array}$$

In the fields of system identification, pattern recognition, etc., because the problem is for a specific system, it is easier to eliminate noisy data; in contrast, in most genetic algorithms, people know very little about the classification discriminant function information, which leads to distinguishing the noise in a large amount of data; it is necessary to avoid overfitting of the data and enhance the generalization ability of the classification algorithm.

(2) $$\begin{array}{c} \mathrm{cov}\left(X\right)=E\left[X\times X^{T}-\left(E\left(X\right)\times E{\left(X\right)}^{T}\right)\right],\\ P\left(S\left(i\right),S\left(j\right),...,S\left(k\right)|T\left(t\right)\right)=P\left(S\left(i\right)|T\left(t\right)\right)\left(S\left(j\right),...,S\left(k\right)|T\left(t\right)\right). \end{array}$$

The method of digital processing of noise in Chinese-English parallel corpus can be in the time domain or in the frequency domain, but the characteristics of the noise of the Chinese-English parallel corpus should be taken into consideration. The noise of Chinese-English parallel corpus is time-varying and can only be regarded as stable in a short period of time. Therefore, the short-term processing technology is the most basic technology to deal with the noise of Chinese-English parallel corpus [20, 21].

(3) $$\begin{array}{c} P\left(B|A\right)=\sum_{i=1}^{N}P\left[B|A\left(i\right)\right]P\left[A\left(i\right)\right],\\ D\left(C\left(1,n\right)\right)=\arg\max\left\{\left(s\left(1,n\right)\right),\left(p\left(1,n\right)\right)\right\}\times P\left(S\left(1,n\right)\right)|\left(C\left(1,n\right)\right). \end{array}$$

If a classification discriminant function is completely local, then the category of each sample point can only be determined by itself, so there is no way to fit or approximate such a function. In fact, it is meaningless to discuss such a discriminant function, because it is given arbitrarily to some extent [22]. The classification method of data mining is to directly or indirectly fit or approximate the piecewise smooth classification discriminant function when the classification discriminant *E*[*f*(*x*)]=∑_*i*=1_^*n*^*w*(*t*) × *f*(*x*(*t*))/∑_*i*=1_^*n*^*w*(*t*) function is unknown.

(4) $$\begin{array}{c} P\left(x\right)=\int P\left[B|A\left(x\right)\right]P\left[A\left(x\right)\right]dA\left(x\right). \end{array}$$

The purpose of estab_l_ishing an acoustic model is to provide an effective method to calculate the distance between the speech feature vector sequence and each pronunciation template. The design of the acoustic model is closely related to the characteristics of language pronunciation. The acoustic model unit size, character pronunciation model, semisyllable model, or phoneme model has a greater impact on the amount of speech training data, system recognition rate, and flexibility. In the training process, after feature extraction and feature dimension compression, using clustering methods or other methods, one or several templates are generated for each pattern category, and the feature vector of the pattern to be recognized is combined with each template in the recognition stage. The similarity is calculated, and then the category is judged.

### 2.2. Genetic Algorithm Network

The concept of genetic algorithm error rate is relatively simple, but when the analytical expression of the class conditional probability density function is more complicated in a multidimensional situation, it is quite difficult to calculate the algorithm complexity. It is precisely because of the importance of algorithm complexity and computational complexity that people have studied some methods of calculating or estimating algorithm complexity when dealing with practical problems. The implicit parallelism and the effective use of global information are two salient features of genetic algorithm. The principle is to replace the original random variable *z* that does not obey the normal distribution with the random variable Y that obeys the normal distribution and then use the second-order moment method to calculate the reliability index. The former enables the genetic algorithm to reflect a large number of areas in the search space by detecting only a small amount of structure, and the latter enables the genetic algorithm to be robust. The genetic algorithm lays a foundation for the use of multilayer feedforward neural networks for efficient learning and improves the overall mining efficiency of the system. However, due to the complexity and diversity of classification mining objects, only relying on the concept of distance as the criterion of the evaluation function may affect the result of feature selection. However, the model has good scalability; as long as some more effective evaluation functions are added, the adaptability of the model will be improved. For specific voice recognition, the opposite is true. The attributes of the object are divided into conditional attributes and decision-making attributes. According to the same attribute value, it is divided into equivalence class. We establish deterministic rules for downlikeness and uncertainty rules (including credibility) for uplikeness, and there are no rules for irrelevant situations. Practice has proved that predictive control has strong robustness and is easy to adjust online. Unfortunately, the mechanism of predictive control's robustness has not yet been theoretically analyzed. This method is often used for attribute reduction.

Figure 2 shows the spatial architecture of the genetic algorithm network. In the genetic algorithm, the training set is first split by attributes (“splitting” along the attributes), a data structure called the attribute list corresponding to the current subset of the training set is established, and the samples in each attribute list are divided by attribute value. Continuous attributes are distributed from small to large attribute values, and discrete attributes are grouped together with the same value. Then, we scan each attribute list to evaluate the Gini index of all the splits of the attribute and take the smallest one as the candidate split. Among all the attributes, the attribute of the candidate split with the smallest Gini index is the split attribute, and we split the training set at the candidate split where the attribute contains the smallest index. First, use the global search ability of genetic algorithm of obtaining the initial weights and thresholds of the BP neural network, so as to prevent the training results of the BP neural network from falling into the local minimum; then, use the samples to train the BP network to obtain the final weights and thresholds. Complete the simulation of the implicit function. The first step in using genetic algorithms to solve this problem is to choose an appropriate solution, because there are three decision variables, each of which can be assumed to be one of two possible values, so each possible business decision for this problem can be naturally expressed as a binary string, where the value 0 or 1 is designated as one of two possible choices. The only information used in the genetic algorithm is the fitness value of the individuals actually appearing in the group. By simulating natural selection and natural genetic processes in the biological world, the genetic algorithm uses genetic operations to transform a group into a new group.  Figure 3 shows a pie chart of the percentages of different data sets based on genetic algorithms. The genetic operation of a simple genetic algorithm is generally composed of three genetic operators: replication, hybridization, and mutation. The copy operator selects and copies the individuals in the current group to the new group with a probability proportional to the fitness value.

If the decision tree is generated completely based on the samples in the training set, then when the sample data has noise, overfitting will occur; that is, the noise is treated as the correct sample and the decision tree is also required to fit. This will actually lead to a decline in the generalization ability of the decision tree and even make the generated decision tree almost unusable. Therefore, the overfitting branch must be pruned. There are two usual pruning methods: one is to use the test set to select the subtree that minimizes the error of the test set, and the other is to use the equivalent MDL (Minimum Description Length) principle for processing. If the output is required to be any continuous function of the input, then use two hidden layers or use different activation functions. Sometimes, even in the case of continuous output, a hidden layer can also meet the requirements, depending on the nature of the valve problem. Note that, in the case of linear separability, the hidden layer is not needed. Because there is no good analytical expression, it can be said that the number of nodes in the hidden layer is directly related to the requirements of the problem, and the number of nodes in the input and output layers. The predictive cepstrum extracted based on the perceptual linear predictive analysis simulates to a certain extent the characteristics of the human ear's voice processing, and some research results in the human ear perceptual perception are applied. Experiments have proved that, with this technology, the performance of the speech recognition system can be improved to a certain extent.

### 2.3. Neural Network Weight Distribution

Neural networks imitate network connection weights. Generally, neural network methods are divided into three types: (1) feedforward network, which is represented by perceptrons, backpropagation models, and functional networks, and can be used for prediction, pattern recognition, and other aspects. (2) Feedback network is represented by discrete model and continuous model of such as field, which are used for associative memory and optimization calculation, respectively. (3) The self-organizing network is represented by the ART model and is used for clustering. Machine learning methods include decision tree method and rule induction method. The former is correspondingly expressed as a decision tree or discriminant tree, and the latter is generally a production rule. The importance sampling method estimates the failure probability by changing the location of the sampling center or sampling random variables with a new probability distribution, so as to reduce the variance of the failure probability estimate and improve the sampling efficiency. The neural network method is mainly the BP algorithm. Its model representation is a forward feedback neural network model (an architecture composed of nodes representing neurons and edges representing connection weights).

Multilayer feedforward neural network is a multilayer neural network system composed of input layer, output layer, and hidden layer. Each layer contains a certain number of neuron nodes.  Table 1 shows the weight distribution of neural network. Generally, in the realization of classification, the number of nodes in the input layer and the output layer is fixed, the nodes in the input layer correspond to the symptom set, and the output nodes represent the mode or state corresponding to the symptom. For multilayer feedforward neural networks, we must first determine several hidden layers. When each node has a different threshold, a hidden layer network can be used to approximate a continuous function in any closed interval, so a three-layer neural network based on the algorithm can complete any mapping.

The topological structure of the feedforward neural network features: information is forwarded without loops. In the feedforward neural network, each layer of neurons only receives the data of the neurons in the previous layer and passes the data to the next layer of neurons after calculation and processing. It solves many problems that are difficult to solve with previous methods.  Figure 4 shows the distributed mapping of neural network units. In the classification process, any decision rule has its corresponding error rate. The error rate reflects the degree of inherent complexity of the classification problem, and it can be considered as a measure of the inherent complexity of the classification problem. After the classifier is designed, the performance is usually measured by the size of the error. Particularly, when designing several different classification schemes for the same problem, the error rate is usually used as the criterion for comparing the quality of the scheme. The decision tree is generated by repeatedly splitting the training set. In each split, a certain split criterion is used to select an attribute, and the training set is divided into multiple subsets (usually divided into two) according to the split criterion, and the corresponding fork of the decision tree is generated at the same time. According to the different uses of the neural network, the output layer of the BP network uses different activation functions: for classification, the Sigmoidal function or the hard extreme function is used; for function approximation, the linear function is used. This process continues until the samples in the subset after the split of the training set corresponding to each current node belong to the same category.

## 3. Results and Analysis

### 3.1. Corpus Noise Data Processing

The acquired dialogue corpus consists of 956 groups of dialogues and 21336 sentences. Manually annotate each sentence in the dialogue with semantics (11 types) and predictions (47 types). In order to use the proposed model for experiments, then 10-fold cross-validation is performed. We have established a GA-BP neural network recognition model, selected training samples and test samples, and extracted the sample moment feature vector as the input of the network and trained and tested the constructed GA-BP network. When the normal random variable Y is used to replace the nonnormal random variable *X*, the cumulative probability distribution function value and the probability density function value at the design checking point x are the same as the original variable. The two types of recognition are compared and analyzed. The network parameters are set to error 0.001, training times to 100, the initial weight of the neural network is set in the range of [−1, 1], and finally the established network is trained and tested. We can see that the GA-BP calculation 50 method has a fast convergence. When the training is 14 times, the set error value has been reached, and the convergence speed of the BP training is not very ideal.  Figure 5 shows the ladder diagram of neural network model training and recognition errors. We use GA to optimize the BP neural network to a satisfactory recognition effect.

Evenly distributed in the test range, the sample information in the test range can be widely learned. In addition, the random number generator is used to directly generate the sample, the range of the sample cannot be selected, and the sample generated by the uniform design can be free to design the value range of the sample. This article uses TensorFlow14.0 to achieve model training, and prediction is completed with sentences as the smallest unit. We set the size of each Word2Vec embedding vector to 100 and the training length to 300 cycles. The best model is found through the mini-batch stochastic gradient descent method. Each mini-batch contains 15 sentences, and the learning rate is fixed at 0.001. The experimental circuit used for the test consists of the following modules: input preamplifier, calibration circuit with a gain adjustment of 0 to 40 dB, linear output attenuator with a step of 5 dB, and SPL with a range of 0 to 100 dB. We apply the genetic algorithm proposed above to optimize the weights or thresholds of the constructed BP neural network. The optimal individual of the network obtained after optimization is decoded, and its value is assigned to the established network, and then the selected training sample extracts moments with the test sample; we use the extracted moment feature vectors as the input of the network and finally analyze the results obtained after simulation. We can see that the recognition rate of the five human gaits using GA-BP neural network is significantly better than that of using BP neural network. It is feasible to use genetic algorithm to optimize the initial weights and thresholds of the network and then to recognize human behavior.

### 3.2. Neural Network Model Simulation

We selected 10,000 sentences containing 6 pronoun sentences in the corpus to exclude the influence of word frequency on the quality of word vectors. Then, in order to simulate the case of low-frequency words, we downsampled the sentences containing the pronoun “you” to 1000, 100, 10, and 5 respectively, and generated word vector representations using the sampled corpus files. Note that different pronouns may appear repeatedly in the same sentence, so the actual sentence size after sampling may not be less than 60,000. This paper combines BP neural network and genetic algorithm, firstly use the global search ability of genetic algorithm of getting the initial weight and threshold of BP neural network training, so as to ensure that the training result of BP neural network will not fall into the local minimum point, and then use samples to train the BP neural network, and finally get a set of weights and thresholds, that is, to complete the simulation of the implicit function. The training algorithm of the word vector uses the model under the Gensim toolkit, the dimension is set to 64, and the rest of the hyperparameters are the default values of the model. It can be seen that when the above 6 pronouns are sampled 20 times at the same time, their relative positions on the two-dimensional plane are relatively concentrated. Near this position, there are common personal pronouns such as “self” and “she.” This shows that the word vectors of personal pronouns are relatively close in the vector space. When the number of samples decreases, the position of the word vector “you” gradually deviates from the gathering position of the pronouns in the space as the number of samples decreases. This shows that the decrease of word frequency will lead to the decrease of the accuracy of its word vector results. If the average position of the 6 pronouns sampled 20 times is regarded as the cluster center and the Euclidean distance is calculated for the word vector, a conclusion consistent with the figure can be obtained.

This paper uses the COAE2014 Task 4 Weibo data set. There are 300 pieces of data in the data set, and 100 of them announce emotional polarity. The experiment uses the data set for word vector training and uses 100 pieces of data published with sentiment polarity for 10-fold cross-validation.  Figure 6 shows the comparison of recall rates of different corpora based on genetic algorithm. In the experimental link, firstly, the sentiment classification effects of different models under random initialization and model are compared, and the corresponding analysis is given. Secondly, on the basis of using the model to initialize the vector, the average F value of each model is compared. This is because the failure domain of the series system is a collection of the failure domains of each function, and the check point of each function is generally on the boundary of the system failure domain. Finally, the semantic expansion scheme proposed in this paper is used on the baseline model to compare the effect of sentiment classification. According to the results, we can see that the four neural network models have obtained better results when using the model to give the initial vector. This is because the model is trained on the corpus of Google News, and the word vector it gives contains the grammatical and semantic information of the text, and this information is lost in the random initialization. Therefore, in subsequent experiments, the Word2Vec model is used for word vector initialization.

Figure 7 shows the histogram of the noise value of the parallel corpus. Since the output has 5 states, it can be described by a 5-bit binary number. The rounding method is adopted here; that is, if the output of the network is less than 0.5, it is considered as 0; otherwise, it is considered as 1. When designing the network in this paper, since there are only 5 types of output, it can be described by a five-digit binary number. It can be seen that the added deep neural network models for unregistered word recognition and concept semantic expansion have improved the F-value of sentiment classification to a certain extent. It proves that the semantic extension model proposed in this article for short texts can effectively improve the accuracy of sentiment analysis.  Figure 8 shows the comparison of the accuracy of parallel corpus noise filtering for different network models.

The neural network method will get two files after segmentation, one is the segmented corpus, and the other is the segmentation dictionary. Each layer of neurons only receives data from the neurons in the upper layer and passes the data to the neurons in the next layer after calculation and processing. In addition to the input layer, each hidden layer and output layer must calculate the received information and all hidden layers and output. The neurons that come out of the layer are called computing nodes. The segmentation dictionary uniquely determines where each word is segmented, so it can be used in other corpora to get the same segmentation results. We apply the English segmentation dictionary on the bilingual corpus to a large-scale monolingual corpus to reduce the impact of the corpus content on word vector training by reducing the size of low-frequency words. Since the neural network algorithm divides by frequency, the position where the English word is disconnected is not necessarily the connection of the root affix. But this method is only to alleviate the problem of data sparseness, and strict segmentation of affix stems is not a necessary condition. There are about 500 affixes in English. The main reason for the sparse data is that the stems of English words may be connected to multiple affixes. According to statistics, after neural network segmentation, the proportion of low-frequency words in both corpora fell below 10%. Aiming at the problem that different corpora may cause deviations in word vector results due to different content or different fields, this paper proposes a seed word vector method to solve the problem. With the help of the subword segmentation results, a word vector with the subword granularity is generated to improve the word vector quality of low-frequency words. The experimental results prove that the subword vector method is indeed effective in transmitting large-scale monolingual corpus information to the translation model for auxiliary training and the accuracy of the translation model can be improved by up to 1.79%.

### 3.3. Analysis of Experimental Results

The experiments in this article use WMT (Workshop on Machine Translation) English-Chinese parallel corpus. We use WMT2017 dev as the verification set and WMT2017 test as the test set. The evaluation of the model translation quality is evaluated by the accuracy script calculation score. In addition, this experiment also uses 700,000 English monolingual corpora collected by the Information and Intelligent Processing Laboratory. In order to reduce the confusion of the model, the above data delete sentences longer than 50. We have conducted word frequency statistics on English words in the corpus. Whether it is a monolingual corpus or a parallel corpus, the proportion of words with a frequency of less than 5 exceeds 70%. This is a very serious data sparse problem, which will directly lead to word vectors. The training result is not ideal. Obviously, in order to improve the quality of word vectors, it is necessary to reduce the proportion of low-frequency words, and the neural network satisfies this demand well. The operands of the neural network need to be set according to language characteristics and corpus size in order to obtain better preprocessing results. This result will be used as the main basis for the experiment. The neural network algorithm segmentation of English words makes the size of the English dictionary plummet and greatly reduces the proportion of low-frequency words in the corpus.

In terms of models, this article uses two current mainstream neural network machine translation models. The cyclic neural network uses the Seq2seq model developed by Google. Its parameters are set to a 4-layer two-way LSTM encoder/decoder. The hidden layer node is 512; batch size is 256. The transformer model uses Google's Tensor2tensor model. Its parameters are set to 6 layers at both ends of the encoder/decoder. The hidden layer nodes are 512 and the batch size is 256. The word vector model uses the FastText model of the Gensim tool. The parameters are set to 512 dimensions of the word vector, the number of windows is set to 5, and the low-frequency word discarding value is 3. The above settings are the default settings of the experiment in this article, and special instructions will be given if there are any changes. The translation evaluation index uses the accuracy script of the Moses tool.  Figure 9 shows the line graph of the accuracy of the word frequency statistics of the parallel corpus. In the comparison model, the model with the highest accuracy value is still the group of Chinese word segmentations first and then neural network segmentations. Compared with the best baseline model, the improvement is 0.72. This shows that the data sparse problem caused by Chinese word segmentation does affect the performance of the translation model and the form of Chinese word segmentation cannot retain the information in Chinese phrases. The above experiment improved the configuration of Chinese word segmentation the most, increasing to 1.52. As the training data increases, the training speed drops quickly. When the training samples increase to a certain level, the network cannot converge to the specified error or reach the specified performance. We believe that this may be due to the word granularity on the Chinese side aggravating the data sparse problem, making it difficult for the model to learn the correspondence between low-frequency words during the training process, and the goal of the subword vector is to alleviate this problem.

In training the topic distribution model, we set the hidden Dirichlet distribution parameter to 0.01. The number of Gibbs sampling is 1000. For efficiency considerations, set *a* = *b* = 0.5. In the short text expansion part, each iteration selects the top 30 terms and concept words to expand the short text.  Figure 10 shows the comparison of corpus data testing accuracy based on genetic algorithm. It can be seen that because the classification algorithm based on concept expansion only expands the original short text by the related concept words, its text classification accuracy has nothing to do with the size of the training set; when the training set is small, the topic model cannot be fully trained, so it cannot be a very good expression of the semantic relationship between concepts and terms, and a certain degree of noise will be added to the semantic expansion. Therefore, when the training set is small, the classification accuracy of the concept expansion model is higher than that of the semantic expansion model. As the size of the training set increases, the algorithm module that uses topic models to mine semantic relevance reflects its superiority. Through the method of dynamic planning, the time distortion of the speech can be adjusted, and the number of training samples has a relatively small impact on the performance of the network. It can also be seen that the recognition rate of easily confused words is low. Because the terminology can express its true meaning explicitly under different topics, the method based on semantic expansion has better accuracy than the method based on concept expansion. The classification accuracy of the mixed model is always better than the two subalgorithm modules. It can be seen that the algorithm model fully expresses the semantic relationship between term words and concept words and effectively expands the short text in terms of conceptualization and semantics.

## 4. Conclusion

In terms of the principles and technology of genetic algorithm, this paper uses genetic algorithm and multilayer feedforward neural network error backpropagation algorithms, such as BP algorithm and conjugate gradient, according to the characteristics of genetic algorithm objects and the characteristics of artificial neural network mining technology. Gradient algorithm, combined with category separability criterion theory, constructed a multilayer feedforward neural network classifier model based on genetic algorithm. This article conducts experiments on the CWMT2018 training set. The experimental results show that the English-Chinese machine translation model with the help of subword vectors as the initialization parameters can increase the accuracy value by 1.79% higher than the baseline model; the English-Chinese neural network machine translation model based on reinforcement learning can increase the accuracy value by 0.6% compared with the baseline model. Without increasing any theoretical difficulties, rolling optimization can easily handle various constraints. It can be applied to large delay, nonminimum phase, and nonlinear systems and obtain better control effects. With data enhancement technology, the translation quality of English-Chinese neural network machine translation improves accuracy by 1.1% compared with the baseline results. The experiment proves that the convergence of GA neural network is better than that of simple neural network and the network is more stable. A comparative analysis of the recognition rate of human behaviors of the two is also done, and the GA neural network can obtain satisfactory recognition results. The model uses the feature selection method proposed in this paper based on the genetic operation and the interclass distance criterion theory to effectively reduce the error of the feature, thus not only focusing on the strong computing power and high accuracy of the multilayer feedforward neural network features, but also improving the efficiency of the classifier as a whole.

## Figures and Tables

**Figure 1:** Hierarchical spatial distribution of multilayer perceptrons.

**Figure 2:** Genetic algorithm network space architecture.

**Figure 3:** Fan chart of the percentages of different data groups based on genetic algorithm.

**Figure 4:** Distributed mapping relationship of neural network units.

**Figure 5:** Neural network model training and recognition error ladder diagram.

**Figure 6:** Comparison of recall rates of different corpora based on genetic algorithm.

**Figure 7:** The histogram of the noise value of the parallel corpus.

**Figure 8:** Comparison of the accuracy of parallel corpus noise filtering by different network models.

**Figure 9:** Line graph of word frequency statistics accuracy of parallel corpus.

**Figure 10:** Comparison of corpus data test accuracy based on genetic algorithm.

**Table 1:** Neural network weight level distribution.

Layer index	Node number	Noise frequency/Hz	Noise amplitude/dB	Weight
1	10	1869	3.19	0.45
2	20	2361	2.48	0.21
3	40	2273	2.31	0.26
4	80	1827	2.96	0.08

## Data Availability

The data used to support the findings of this study are available from the corresponding author upon request.
